The article "Robust Blood Cell Image Segmentation Method Based on Neural Ordinary Differential Equations" was published in 2021. Journal: Comput Math Methods Med.

# Robust Blood Cell Image Segmentation Method Based on Neural Ordinary Differential Equations

**DOI:** 10.1155/2021/5590180

**Published:** 2021-08-07

**Authors:** Dongming Li, Peng Tang, Run Zhang, Changming Sun, Yong Li, Jingning Qian, Yan Liang, Jinhua Yang, Lijuan Zhang

**Affiliations:** ^1^School of Information Technology, Jilin Agricultural University, Changchun 130118, China; ^2^College of Opto-Electronic Engineering, Changchun University of Science and Technology, Changchun 130022, China; ^3^College of Computer Science and Engineering, Changchun University of Technology, Changchun, Jilin 130012, China; ^4^CSIRO Data61, Epping, NSW 1710, Australia

## Abstract

For the analysis of medical images, one of the most basic methods is to diagnose diseases by examining blood smears through a microscope to check the morphology, number, and ratio of red blood cells and white blood cells. Therefore, accurate segmentation of blood cell images is essential for cell counting and identification. The aim of this paper is to perform blood smear image segmentation by combining neural ordinary differential equations (NODEs) with U-Net networks to improve the accuracy of image segmentation. In order to study the effect of ODE-solve on the speed and accuracy of the network, the ODE-block module was added to the nine convolutional layers in the U-Net network. Firstly, blood cell images are preprocessed to enhance the contrast between the regions to be segmented; secondly, the same dataset was used for the training set and testing set to test segmentation results. According to the experimental results, we select the location where the ordinary differential equation block (ODE-block) module is added, select the appropriate error tolerance, and balance the calculation time and the segmentation accuracy, in order to exert the best performance; finally, the error tolerance of the ODE-block is adjusted to increase the network depth, and the training NODEs-UNet network model is used for cell image segmentation. Using our proposed network model to segment blood cell images in the testing set, it can achieve 95.3% pixel accuracy and 90.61% mean intersection over union. By comparing the U-Net and ResNet networks, the pixel accuracy of our network model is increased by 0.88% and 0.46%, respectively, and the mean intersection over union is increased by 2.18% and 1.13%, respectively. Our proposed network model improves the accuracy of blood cell image segmentation and reduces the computational cost of the network.

## 1. Introduction

One of the most basic methods to diagnose diseases is by examining the blood smear through a microscope to check the shape, number, and proportion of red blood cells and white blood cells. However, manual examination of a blood microscope image is a time-consuming and laborious task. In recent years, with the development of computer vision and medical image processing technology, the recognition of medical microscopic cell images has also made considerable progress in the field of medical image processing. The research on medical image processing methods has become an important research direction in image processing and analysis.

The article "Robust Blood Cell Image Segmentation Method Based on Neural Ordinary Differential Equations" was published in 2021. Journal: Comput Math Methods Med.

Image segmentation is an important stage in the process of image analysis and processing. Traditional medical image segmentation methods mainly include activity contour, intensity thresholding, mathematical morphology, region growing, and watershed algorithm [1–5]. Since the fully convolutional neural network (FCN) [6] was first proposed by Long et al., it has achieved semantic segmentation of natural images from end to end, and it has also indicated the most progressive capacity in image segmentation. And they regard FCN as a foundation and have innovated tremendous numbers of excellent semantic segmentation networks [7] from different perspectives under the stimulation from all kinds of semantic segmentation challenging competitions. Ronneberger et al. [8] focused on the large size and small quantity of medical images, providing a U-Net network model which adopted a coding-decoding structure. After 4 times of pooling during downsampling, dimensional splicing and fusion are performed with the corresponding scale in upsampling for adding feature information. To construct the pixel weight matrix, the closer it is to the cell's boundary, the larger the pixel weights will be, so it would be trained specifically. Kowal et al. [9] combined a convolutional neural network (CNN) and a seeded watershed algorithm [4] to segment the nucleus in breast cancer cell images, utilizing the accurate nucleus mask produced by CNN to replace the nucleus mask which was defined by normal thresholding. This process generates watershed topographic maps and nucleus seeds, and then, a watershed algorithm was used to separate the overlapping nucleus. Song et al. [10] proposed a multiscale convolutional network (MSCN) and a method based on image partition segmentation of the cervical cytoplasm and nucleus. They extracted features by MSCN and then divided the central region of each pixel. This method can segment all the nuclei in the cell images, but it could not distinguish normal cells and abnormal cells. Araújo et al. [11] used CNN to segment abnormal cells and blocky abnormal cells with high image overlap from digital images of conventional pap smears, filtering input images and eliminating cells that only include background or bad information. They adopted postprocessing to improve segmentation of abnormal cells and sorted the images according to probability of containing abnormal cells in the image. Öztürk et al. [12] proposed a new DCNN structure based on the residual network (ResNet) [13] and the deconvolutional network [14] structure. Semantic segmentation would be launched according to histopathological cell type, and all nuclei would be identified. They were classified as cancerous or normal according to each cell type. Shibuya and Hotta [15] proposed the feedback U-Net [8] network based on convolution long-short-term memory (LSTM). The output of U-Net reports back to the input, and then, it is fed into the second round. They extracted second-round features based on the first-round features by utilizing convolution LSTM [16]. Convolution LSTM that is used to process ordered data is a convolutional version of LSTM [17]. Chen et al. [18] proposed a new neural network that is referred to as neural ordinary differential equations (NODEs). This paper refers to the idea of Chen et al. [18]. We used the latest NODEs to improve the classic medical image segmentation method based on the U-Net network.

The article "Robust Blood Cell Image Segmentation Method Based on Neural Ordinary Differential Equations" was published in 2021. Journal: Comput Math Methods Med.

We put an ODE-block into a U-Net network model for blood cell image segmentation (named NODEs-UNet). The proposed NODEs-UNet network model can effectively reduce the use of parameters and improve the segmentation effect. NODEs can adapt to the receptive fields (RFs). There is no need to optimize the RFs for various segmentation tasks, and we only need to adjust the error tolerance of ODE-block. The generalization ability of the NODEs-UNet model architecture is strong.

## 2. Image Preprocessing

The experiment dataset in this paper was provided by the Center for Medical Image and Signal Processing (MISP) and the Department of Pathology, Isfahan University of Medical Sciences [19]. MISP.rar contains 148 clear blood cell smear images with a size of 775 × 519 pixels. Since the blood cell image is quite large, we picked up appropriate areas for convenient network training. We cropped 100 blood cell images with a size of 256 × 256 pixels by selecting a suitable area. To ensure the accuracy of the training model, we retained 20 images as the testing set and we used the remaining 80 images to increase the dataset to 800 by data augmentation. Besides, we used a ratio of 3 : 1 as the training set and the validation set. The image label was obtained by manual labeling by using the labeling tool LabelMe. There are three cell types that need labeling: background, white cells, and red cells. They are given the labels of 0, 1, and 2, respectively.  Figure 1 shows the original blood cell image and its postvisualization of labels.

The article "Robust Blood Cell Image Segmentation Method Based on Neural Ordinary Differential Equations" was published in 2021. Journal: Comput Math Methods Med.

This paper employed blood smear images, which contain a small number of white blood cells and a large number of red blood cells. The original blood cell images are in color, and we use the color image for segmentation. We conducted preprocessing to the cell image and enhanced the contrast among cell images for segmenting the targets better. The blood cell images were converted from the RGB color space to the YUV space. The pseudocode is as follows:

Img = Read(Path)

Y,U,V = BGR2YUV(Img)

Y´ = clahe_equalized(Y)

Img = YUV2BGR(Y´,U,V)

where “Y” means brightness. “U” stands for the difference between the blue channel and brightness. “V” means the difference between the red channel and brightness.  Figure 2 shows the original cell image and the preprocessed image.

## 3. Methodology

We present a novel segmentation method based on neural ordinary differential equations (NODEs) and U-Net for blood cell image segmentation. Firstly, the NODEs are introduced. Then, based on the classic U-Net network, we imported an ODE-block into the U-Net network architecture and determined the ODE-block location in the network. Finally, the proposed NODEs-UNet network architecture is built. The segmented image is constructed based on the NODEs-UNet network framework.

### 3.1. Neural Ordinary Differential Equation

Neural ordinary differential equation means a differential equation with a single independent variable. We are supposed to find the general solution of the unknown *f*(*x*) for an ordinary differential equation normally. For instance, the general solution of equation *f*′(*x*) = 2*x* is *f*(*x*) = *x*^2^ + *C*, where *C* means an arbitrary constant. But the more common method to solve this problem in practice is by using an ODE-solver. That is, given an initial value *f*(*x*_0_), this does not have to find the general solution of *f*(*x*) when seeking the unknown value *f*(*x*_1_) except approaching its value gradually. In terms of the neural network, they are similar to an extreme complicated composite function whether they are a fully connected network, recurrent network, or convolutional network. The number of compositions is equal to the depth of the layers. For instance, a two-level fully connected network could be

(1) $$\begin{array}{c} h_{t+1}=f\left(h_{t},\theta_{t}\right),\\ h_{t+2}=f\left(h_{t+1},\theta_{t+1}\right),\\ h_{t+2}=f\left(f\left(h_{t},\theta_{t}\right),\theta_{t+1}\right), \end{array}$$

where *h*_*t*_ is the input value of the hidden unit of the *t*-th layer and *f* parameterizes the neural network by *θ*_*t*_. Therefore, every neural network layer is similar to a universal function approximator.

The article "Robust Blood Cell Image Segmentation Method Based on Neural Ordinary Differential Equations" was published in 2021. Journal: Comput Math Methods Med.

A residual network (ResNet) [13] is a special type of convolutional network. It solved the gradient reversion problem with residual connection, which means that the gradient can still be effectively transmitted back to the input end when the neural network layer is very deep.  Figure 3 is the structure of a ResNet-block. The output of the ResNet-block combines the input information and the output information of the internal convolution operation. This residual connection ensures that the accuracy of the deep model is at least not lower than the accuracy of the shallow network.

We can illustrate the ResNet-block above formally as an equation below: *h*_*t*+2_ = *h*_*t*_ + *f*(*f*(*h*_*t*_, *θ*_*t*_), *θ*_*t*+1_), which stands for the whole ResNet-block above. If we rewrite it in the form of a residual network, that is,

(2) $$\begin{array}{c} h_{t+2}=h_{t}+f\left(f\left(h_{t},\theta_{t}\right),\theta_{t+1}\right). \end{array}$$

We can find that the traditional neural network *f* is directly parameterized as hidden layers and the residual neural network *f* parameterizes the residual among hidden layers. But the neural ordinary differential equation in this paper takes another way to use for parameterizing the derivative in hidden states by the neural network. By assuming the discrete layers as continuous layers and parameters, this continuous transformation form can be expressed as a neural ordinary differential equation (NODE):

(3) $$\begin{array}{c} \frac{dh\left(t\right)}{dt}=f\left(h\left(t\right),t,\theta \right), \end{array}$$

where *f* is defined as a neural network as before, but now this and its parameter *θ* are a unit, and *t* is also fed into the neural network as an independent parameter. From the perspective of derivative definition, when the change of *t* tends to become infinitely small, the change of the hidden state *dh*(*t*) can be modeled by the neural network. When *t* changes slowly from the initial to the end, the change of *h*(*t*) ultimately represents the result of forward propagation. In this way, using the neural network to parameterize the derivative of the hidden layer, the neural network layer is indeed continuous.

If the numerical solution of the ordinary differential equation can be obtained, then it is equivalent to forward propagation. Now, we convert equation (3) to

(4) $$\begin{array}{c} \int_{t_{0}}^{t_{2}}dh\left(t\right)=\int_{t_{0}}^{t_{2}}f\left(h\left(t\right),t,\theta \right)dt, \end{array}$$

(5) $$\begin{array}{c} h\left(t_{2}\right)=h\left(t_{0}\right)+\int_{t_{0}}^{t_{2}}f\left(h\left(t\right),t,\theta \right)dt. \end{array}$$

From equation (5), we can see that the numerical solution of ODE *h*(*t*_2_) requires the integral of the neural network *f* from *t*_0_ to *t*_2_. It is a problem about the initial value of ODE. We can obtain the result with an ODE-solver directly. Such an ODE-solver can also control the numerical error so that we can make a contrast between computing ability and model accuracy.  Figure 4 is the structure of the ODE-block.

The article "Robust Blood Cell Image Segmentation Method Based on Neural Ordinary Differential Equations" was published in 2021. Journal: Comput Math Methods Med.

### 3.2. The Location of ODE-Block

The network architecture of this paper is based on the classic U-Net fully convolutional neural network model in medical image segmentation. Considering the reduction of the computational cost, we decrease the number of convolutional cores in the convolution layers to a half in the original U-Net network. In order to study the influence of a single ODE-block on the network at different positions, we imported an ODE-block in the U-Net network architecture which is shown in Figure 5. The training set, validation set, and testing set of the whole networks are consistent, and the error tolerance of the ODE-block solver is 1*e*^−3^. When we train the network, we input the training set and the validation set, and the training times (epochs) are 50 times. We use a callback function to save the network model with the minimum val_loss of the validation set.

Nine ODE-blocks obtained in the above experiment were tested on the testing set. The cell image segmentation results were evaluated by pixel accuracy (PA), class pixel accuracy (CPA), mean intersection over union (MIoU), and computation time, and the comparison results are shown in Table 1.

From Table 1, we can see that compared with the U-Net network and the nine ODE-block-based networks, it can be seen that after the ODE-block is added, the PA and MIoU have been significantly improved. The computation time is obviously surging, which is the time it takes for the network to segment twenty blood cell images. Compared with the nine ODE-block-based networks, the location where the ODE-block is added has no obvious impact on PA and MIoU, but it has a greater impact on the computation time, so we could conclude that the location where the ODE-block is added goes down as the U-Net “U”-shaped structure goes down. And the time is much shorter when the “U”-shaped structure keeps going down. The more the “U”-shaped structure goes up, the longer the time is.

### 3.3. NODEs-UNet Neural Network

In this paper, we present a novel blood cell image segmentation method based on NODEs and U-Net (named NODEs-UNet) neural network framework. It is based on the U-Net network model, and downsampling is performed through the maximum pooling layer. For the coding part, each time it passes through a pooling layer, a new scale is constructed, and there are five scales including the original image. Finally, the convolution results in five scales are fused. The convolutional layer extracts features, and the “same” convolution is used to keep the image size unchanged before and after convolution. Upsampling is performed through bilinear interpolation, and the scale corresponding to the feature extraction part is fused with each upsampling.

The article "Robust Blood Cell Image Segmentation Method Based on Neural Ordinary Differential Equations" was published in 2021. Journal: Comput Math Methods Med.

From Section 3.2, it can be concluded that the ODE-block location that is added goes down with the U-Net “U”-shaped structure, and the time is shorter. Therefore, we add one ODE-block with error tolerance l*e*^−6^ and two ODE-blocks with error tolerance l*e*^−4^ at the bottom of the “U” shape, as shown in Figure 6.

The final prediction result of this network uses the activation function softmax, that is,

(6) $$\begin{array}{c} a=\text{Softmax}\left(z_{i}\right)=\frac{e^{z_{i}}}{\sum_{c=1}^{C}e^{z_{c}}}, \end{array}$$

where *z*_*i*_ is the output value of the *i*-th node and *C* is the number of output nodes which is the number of classification categories. The output of the multiclass is converted into a probability distribution in the range of [0, 1] through the softmax function, which means the probability that node *i* belongs to the background, white cells, or red cells. We use categorical cross entropy as the loss function of the network, which is often suitable for multiclass problems and can avoid the problem of reduced learning rate of the mean square error loss function. The equation is as follows:

(7) $$\begin{array}{c} \text{loss}=-\frac{1}{n}\left(y\ln a+\left(1-y\right)\ln\left(1-a\right)\right), \end{array}$$

where *y* is the probability distribution of the expected output and *a* is the probability distribution of the actual output of the network. When the value of the cross entropy is smaller, the two probability distributions are closer.

## 4. Experimental Results and Discussion

The proposed NODEs-UNet network framework was applied to the problem of multiclass blood cell image segmentation, and it is used to evaluate the role of exploiting the ODE-block in segmentation. The real image dataset was chosen from the publicly available dataset on MISP and the Department of Pathology, Isfahan University of Medical Sciences, that contains blood smear microscopic images with red cells and white cells, namely, the MISP01 dataset [19]. The results of this experiment were compared with those of the U-Net network [8] and the ResNet network [13]. The reason we choose these two networks is that the U-Net network is good at semantic segmentation and it is the basis of our proposed NODEs-UNet network. The ResNet network is also based on the reduced version of the U-Net network in this paper, and the residual module is added to the U-Net network. The added ResNet-block location was referred to the D-LinkNet [20] architecture; then, we built the ResNet network model. In the following sections, we give the experimental settings. Then, we compare our method with those two methods and give the statistical results.

The article "Robust Blood Cell Image Segmentation Method Based on Neural Ordinary Differential Equations" was published in 2021. Journal: Comput Math Methods Med.

### 4.1. Experimental Settings

In this study, all the experiments are implemented in a Ubuntu 16.04 LTS 64-bit operating system with Intel Xeon E5 64 core CPU and NVIDIA GeForce GTX 1080 Ti 11 G ∗ 4 GPU, based on the Keras deep learning framework equipped with the NODEs-UNet network model. The ODE-block uses TensorFlow. We complete the training and testing for blood cell image segmentation in CUDA 8.0 GPU calculating the platform and cuDNN 7.5 deep learning GPU acceleration library.

In order to increase the training speed, we call the function multi_gpu_model() to copy the model on four GPUs. Each GPU calls its own model, running on its own dataset, and then connects all the running results together. In order to avoid memory overflow, the model is built on the CPU. We input the training set and validation set to train the network, saving the model with the smallest loss (val_loss) in the validation set in a single model and saving the network framework in a HDF5 file.

### 4.2. Validation on Blood Cell Image Segmentation

For the MISP01 dataset, four randomly selected blood cell images were used for blood cell image segmentation based on the NODEs-UNet framework, and Figure 7 shows the results.  Figure 7(a) is the original blood cell images.  Figure 7(b) is the preprocessed blood cell images using an adaptive histogram equalization method (see Section 2).  Figure 7(c) is the corresponding labels of blood cell images.  Figure 7(d) is the segmentation result using our proposed algorithm. From Figure 7, we can see that our method can accurately segment background, red cells, and white cells. It has clear boundary and complete details, and the segmentation results are very close to the ground truth.

In order to further verify our proposed segmentation method based on the NODEs-UNet network in this paper, we compared and analyzed the quality of the segmentation results from our method with the related works developed on the basis of the U-Net network [8] and the ResNet network [13], and the comparison on the segmentation results are shown in Figure 8. Figure 8 shows four randomly selected blood cell image segmentation results using three networks. As shown in Figure 8(a), the original blood cell images are randomly selected from the MISP01 dataset [19] with blurring and noise.  Figure 8(b) is the enhanced cell images using an adaptive histogram equalization method (Section 2).  Figure 8(c) is their corresponding ground truth.  Figure 8(d) shows the segmentation results after applying U-Net to the images.  Figure 8(e) is for the segmentation result after applying ResNet to the images. As shown in Figure 8(f) for the result of our proposed segmentation method based on the NODEs-UNet network, we can see that our work can provide more accurate segmentation and more details.

The article "Robust Blood Cell Image Segmentation Method Based on Neural Ordinary Differential Equations" was published in 2021. Journal: Comput Math Methods Med.

To quantitatively measure and compare the accuracy of our proposed method with other methods, we applied each of the methods on the segmented dataset and compared it with the ground truth. Then, we counted the truly and falsely detected segmentation results. Effectiveness measures based on PA, CPA, and MIoU are calculated.  Table 2 shows the evaluation results of each method on the blood cell image segmentations for the testing set, where parameter *M* refers to the memory space occupied by the parameter weight of the network model. Figures 9 and 10 show the specific PA and MIoU indicators of the segmentation results of each network in 20 blood cell images.

Observing Table 2, by comparing the objective evaluation data (PA, CPA, and MIoU) of the U-Net network with those of the ResNet and NODEs-UNet networks, we concluded that on the basis of the U-Net network architecture, whether by adding the ResNet-block or the ODE-block, both segmentation results are significantly improved. For the ResNet network, the PA and MIoU have increased by 0.42% and 1.05%, respectively, and the PA and MIoU of the NODEs-UNet network increased by 0.88% and 2.18%, respectively. This is mainly because the output of the ResNet-block and the ODE-block combines the input information with the output information of the internal module operation, and this connection method ensures that in the network model after being added, the accuracy of the module is at least not lower than the accuracy of the initial network model. And due to the limitation of the computational power of the experimental equipment, the number of convolution cores in the convolutional layer in the U-Net network in this paper is twice as small as that in the traditional U-Net network, and the complexity is lower. After adding the ODE-block, the depth of the network is increased, so the accuracy of the network is significantly improved.

Then, by comparing the indicator data (PA and MIoU) of the NODEs-UNet network and the ResNet network, it can be seen that the ODE-block has more advantages in performance than the ResNet-block, and the PA and MIoU in the NODEs-UNet network has increased by 0.46% and 1.13%, respectively, as compared to those in the ResNet network. This is because the residual network is a special case of ordinary differential equations, which is the discretization of Euler's method. Euler's method is very intuitive for solving ordinary differential equations, that is, *h*(*t* + Δ*t*) = *h*(*t*) + Δ*t* × *f*(*h*(*t*), *t*). Whenever the hidden layer takes a small step Δ*t* along *t*, the new hidden layer state *h*(*t* + Δ*t*) should take a small step in the existing direction. If we walk from *t*_0_ to *t*_1_ in such a small step, then the numerical solution of ODE is obtained. If Δ*t* is equal to 1 every time, then the Euler method of discretization is equal to the expression of the residual module *h*(*t* + 1) = *h*(*t*) + *f*(*h*(*t*), *t*). But Euler's method is a basic method adopted to solve ordinary differential equations. Each step will make a little error, and the error will be accumulated.

The article "Robust Blood Cell Image Segmentation Method Based on Neural Ordinary Differential Equations" was published in 2021. Journal: Comput Math Methods Med.

The ODE-solver in the NODEs-UNet network does not move a fixed step length like Euler's method. It will select an appropriate step length to approximate the real solution according to the given error tolerance. Reducing the error tolerance will increase the number of evaluations of the function, similar to increasing the depth of the model. Therefore, we can change the behavior of the neural network by changing the error tolerance. During training, the error can be reduced, the accuracy rate can be improved, and a better neural network can be learned. During testing, the error can be increased according to the actual computing environment, the number of function evaluations can be reduced, and we can obtain the segmentation result faster. By comparing the memory space occupied by the NODEs-UNet network with the ResNet network parameters, the memory space occupied by the NODEs-UNet network is only 46% of the ResNet network. This is due to the derivative of the parameterized hidden state of the ODE-block, which similarly constructs continuity layers and parameters. There are no intermediate results stored in the forward propagation process, so it only needs approximately constant memory cost.

## 5. Conclusion

This paper combines the neural ordinary differential equation with the U-Net network to segment blood smear images. Compared with the more common semantic segmentation using fully convolutional networks, this paper does not improve on feature extraction and multiscale fusion, but it is directly based on the U-Net network model. The ODE-block is added to improve the network and improve the network accuracy for cell image segmentation. Utilizing the characteristics of the ODE-block, we use the ODE-solver in the ODE-block to parameterize the derivative of the hidden state, instead of directly parameterizing the hidden state as usual. This connection method can achieve the same effect as the residual network and can effectively avoid the problem of network degradation in the deep network. Of course, the network layer of this paper is not very deep, and the advantages of this paper have not been fully utilized. The ODE-block can select an appropriate step length to approximate the real solution according to the given error tolerance. Based on these characteristics, reducing the error tolerance will increase the number of evaluations of the function, which is similar to increasing the depth of the model without increasing the parameters of the model. We reduce the error tolerance of the ODE-block in the condition of limited computing resources, and a deep network model can also be built.

The article "Robust Blood Cell Image Segmentation Method Based on Neural Ordinary Differential Equations" was published in 2021. Journal: Comput Math Methods Med.

The next research plan is to perform convolution with a 1 × 1 convolution kernel for each scale sampled on the NODEs-UNet network. We will perform multiscale fusion of all outputs, connect them to the fully connected layer, and do linear regression. So we can directly output the number of white blood cells and red blood cells in the blood image.

## Figures and Tables

**Figure 1:** Display of an example image and its labels: (a) a blood cell image; (b) corresponding label shown in color.

**Figure 2:** Blood cell image preprocessing: (a) original blood cell image; (b) preprocessed cell image.

**Figure 3:** Structure of a ResNet-block.

**Figure 4:** Structure of ODE-block.

**Figure 5:** Nine different ODE-block locations.

**Figure 6:** NODEs-UNet neural network framework.

**Figure 7:** Blood cell image segmentation results: (a) original blood cell images; (b) preprocessed blood cell images; (c) corresponding labels; (d) segmentation results by our algorithm based on the NODEs-UNet network.

**Figure 8:** The original images and the comparison results based on three networks on the MISP01 dataset: (a) original image; (b) preprocessed blood cell image; (c) ground truth; (d) segmented method based on the U-Net network; (e) segmented images based on the ResNet network; (f) results from our proposed method based on the NODEs-UNet network.

**Figure 9:** Experimental results for the PA index.

**Figure 10:** Experimental results for the MIoU index.

**Table 1:** Comparison results of different ODE-block positions.

Algorithm	PA (%)	CPA (%)			MIoU (%)	Time (s)
		Background	Red cells	White cells		
U-Net	94.59	92.55	96.54	94.10	88.58	0.15
ODE-UNet1	95.05	94.25	95.97	93.92	89.80	7.35
ODE-UNet2	95.08	94.23	95.69	95.98	89.68	3.73
ODE-UNet3	95.11	95.14	95.70	91.65	89.61	1.94
ODE-UNet4	95.19	94.08	96.51	93.42	90.17	1.03
ODE-UNet5	95.05	95.62	94.62	94.53	89.62	0.61
ODE-UNet6	95.14	93.78	96.34	95.39	90.09	1.06
ODE-UNet7	95.17	93.80	96.59	94.19	90.02	1.95
ODE-UNet8	95.16	94.33	96.30	92.98	89.91	3.72
ODE-UNet9	95.14	94.33	96.23	93.15	90.03	7.35

The article "Robust Blood Cell Image Segmentation Method Based on Neural Ordinary Differential Equations" was published in 2021. Journal: Comput Math Methods Med.

**Table 2:** Comparison results for three networks.

Algorithm	PA (%)	CPA (%)			MIoU
		Background	Red cells	White cells	
U-Net	94.42	92.55	96.54	94.10	88.43
ResNet	94.84	94.55	95.60	92.89	89.48
NODEs-UNet	95.30	94.58	95.94	95.37	90.61

## Data Availability

The source code supporting the study will be available from the corresponding author upon reasonable request.
